# Fault Diagnosis in Regenerative Braking System of Hybrid Electric Vehicles by Using Semigroup of Finite-State Deterministic Fully Intuitionistic Fuzzy Automata

**DOI:** 10.1155/2022/3684727

**Published:** 2022-04-22

**Authors:** Sajida Kousar, Farah Aslam, Nasreen Kausar, Dragan Pamucar, Gezahagne Mulat Addis

**Affiliations:** ^1^Department of Mathematics and Statistics, International Islamic University Islamabad, Islamabad, Pakistan; ^2^Department of Mathematics, Faculty of Arts and Sciences, Yildiz Technical University, Esenler 34210, Istanbul, Turkey; ^3^Department of Logistics, University of Defence in Belgrade, Belgrade, Serbia; ^4^Department of Mathematics, University of Gondar, P.O. Box: 196, Gondar, Ethiopia

## Abstract

Regenerative braking is one of the most promising and ecologically friendly solutions for improving energy efficiency and vehicle stability in electric and hybrid electric cars. This research describes a data-driven method for detecting and diagnosing issues in hybrid electric vehicle regenerative braking systems. Early fault identification can help enhance system performance and health. This study is centered on the construction of an inference system for fault diagnosis in a generalized fuzzy environment. For such an inference system, finite-state deterministic fully intuitionistic fuzzy automata (FDFIFA) are established. Semigroup of FDFIFA and its algebraic properties including substructures and structure-preserving maps are investigated. The inference system uses FDFIFA semigroups as variables, and FDFIFA semigroup homomorphisms are employed to illustrate the relationship between variables. The newly established model is then applied to diagnose the possible fault and their nature in the regenerative braking systems of hybrid electric vehicles by modeling the performance of superchargers and air coolers. The method may be used to evaluate faults in a wide range of systems, including autos and aerospace systems.

## 1. Introduction

Complex processes and phenomena are prevalent in modern science and technology, about which comprehensive knowledge is not always accessible. Mathematical models are created to address many types of systems having aspects of uncertainty in such instances. A substantial portion of these approaches is built on the so-called fuzzy sets, which are a new extension of conventional set theory. The fuzzy set proposed by Zadeh [1] is based on the formulation of membership function from *X* to [0,1], where the images are termed as membership grades or degrees of membership of elements of *X*. Atanassov [2] proposed the notion of an intuitionistic fuzzy set (IFS), which is an extension of the perception of the fuzzy set where the degree of nonmembership is also considered along with the degree of membership. A finite-state machine (FSM) or finite-state automata (FSA) are a mathematical model of computation that can be changed from one state to another state in connection to suitable inputs. There are two types of FSMs, deterministic FSM (DFSM), the one who accepts or rejects a given string of inputs, following a state sequence uniquely obtained from the string, and nondeterministic FSM (NDFSM), which does not obey these restrictions. Moreover, for each NDFSM an equivalent DFSM can be constructed. Fuzzy automata are used to handle system uncertainties more accurately, whereas classical automata fail to cater to the circumstances. Fuzzy automata have been frequently employed since the introduction of fuzzy technology and neural networks [3–13]. Furthermore, there were a variety of problems to be resolved, for example, medical diagnosis, car anti-crash radar, freeway management, urban road traffic control, and obstacle recognition in front of a vehicle, which required flexible, quick, and accurate decisions, and then, fuzzy neural network automata (FNNA) [14–17] are an excellent choice. FNNA had an increasingly prominent role, particularly in data communications. In FNNA, fuzzy technology is used to compare ordinary identification and control devices using several features and techniques of the neural network including fast and accurate numerical calculation of large numbers and self-organization learning ability. As a result, FNNA was able to solve a variety of problems in a flexible, quick, and precise manner and it had several advantages such as compact size, lightweight, and stability. The research findings also revealed that it has a significant ability for self-organization learning and the experimental results demonstrated fuzzy automata's superiority. Li and Qiu [18] introduced the technique of minimizing fuzzy automata and constructed a new automaton system that dealt accurately with many states at a time. They used an ordered lattice to reduce a fuzzy automaton of *n* states to another fuzzy automaton with *m* states (*m* < *n*) that were functionally correspondent to the original fuzzy automata. Several language-preserving methods for minimizing deterministic fuzzy automata were established. Moghari and Zahedi's [19] method preserves both language and structure in minimization process. De Mendivil and Garitagoitia [20] described the factorization of fuzzy states that are used in the determination of fuzzy automata. Stamenkovic et al. [21] studied fuzzy automata and reduction in fuzzy automaton states and relational equations of the fuzzy system by considering the solution of the fuzzy equivalent equation. These solutions are then used to reduce the number of acceptable states. The solution of the fuzzy system of quasi-order number was also used to reduce the states of the fuzzy automaton.

The relationship between semigroup and FSA was established by Krohn and Rhodes' [22] discussed semigroup decomposition employing decomposing of FSA. A semigroup is an important algebraic structure, which serves as the theoretical foundation for a variety of scientific fields with several applications [23]. Semigroup's role in theoretical computer science is inevitable; in particular, semigroup and automata are widely studied and applied in artificial intelligence, game theory, dynamical system, system biology, and fault diagnosis. During the investigation, it was discovered that to diagnose a machine's problem situation, it is necessary to look at its operating state, fault degree, accuracy degree, and expected changes between states at different stages, which can be done by establishing an appropriate FSA. The uncertainty and ambiguity in the diagnostic process enforce to carry out the mathematical computation in a fuzzy environment. A semigroup of finite deterministic intuitionistic fuzzy automata (FDIFA) is used to detect default in any machine [24] by identifying its crucial components, and it can perform characteristic processing using its state transition mapping. Furthermore, because it accurately and efficiently detects the fault, the maximum value of the membership and nonmembership grades can be used to diagnose the maximum default and current running state of any machine. Membership and nonmembership grades can be assigned based on the nature and seriousness of the fault. The algebraic properties of FDIFA semigroup are employed in the formulation of inference systems over FDIFA semigroup. Fuzzy inference is a method of formulating a rule or a mapping from a given set of inputs to a given set of outputs utilizing fuzzy logic. The fuzzy inference system is widely used in control systems [25], artificial intelligence [26, 27], decision-making [28], forecasting [29], and game theory [30]. Fuzzy set over a non-empty set *X* as defined by Zadeh is a function (membership function) from *X* to the closed interval [0,1] so the representation of uncertain data using closed interval is equivalent to representation using fuzzy sets [31, 32]. The fuzzy inference of fuzzy automata is introduced and utilized in machine defect diagnosis as the impact of combination of fuzzy automaton rules and method of fuzzy set is greater than the classical automata. For the derivation of automata, some researchers used neural networks [33, 34]. Although neural networks and fuzzy systems are not the same, fuzzy inference has been widely applied in the disciplines of control and intelligence [35]. The fuzzy inference system and fuzzy automata and algebraic structures on fuzzy automata are investigated and successfully applied in computer science and engineering [36]. A intuitionistic fuzzy set is a very useful generalization of fuzzy set, which provides an effective framework to handle imprecision and uncertainties more accurately than the fuzzy set and logic. This motivates us to incorporate the concept of nonmembership grades in fuzzy automata. The work is based on the development of inference systems and automata in an intuitionistic fuzzy environment. Intuitionistic fuzzy automata have several states at a certain time or stage, each equipped with a certain grade of reliability and non-reliability. Thus, the intuitionistic fuzzy automata are more realistic and close to the objective. To achieve the goal, finite-state deterministic fully intuitionistic fuzzy automata (FDFIFA) are defined in Section 2. In Section 3, monoid on fully intuitionistic fuzzy automata is designed and its algebraic properties are investigated, and intuitionistic fuzzy inference rules on FDFIFA monoids are established in Section 4. In Section 5, the mathematical computations are supported and justified by conduction fault diagnosis in hybrid vehicle regenerative braking system in application (see Figure 1).

## 2. Fully Deterministic Finite-State Intuitionistic Fuzzy Automata

The sixfold AT=(*T*, *I*(*T*), *ϑ*, *s*_*i*_, *E*, *G*) is referred to as a fully deterministic finite-state intuitionistic fuzzy automata (FDFIFA) in which *s*_*i*_ ∈ *I*(*T*) is the initial state; *T* is a finite family of states; *I*(*T*) is an intuitionistic fuzzy subset of states with grade of membership *μ* : *T*⟶(0,1] and grade of nonmembership *ν* : *T*⟶[0,1); *E* is a finite family of input letters/symbols; *G* is an intuitionistic fuzzy set of terminal/accepting states with *G*⊆*I*(*T*); and *ϑ* : *I*(*T*) × *E*⟶*I*(*T*) is the transitional mapping with *ϑ*((*t*_*i*_, *μ*^*t*_*i*_^, *ν*^*t*_*i*_^), *e*)=(*t*_*j*_, *μ*^*t*_*j*_^, *ν*^*t*_*j*_^), where (*t*_*i*_, *μ*^*t*_*i*_^, *ν*^*t*_*i*_^), (*t*_*j*_, *μ*^*t*_*j*_^, *ν*^*t*_*j*_^) ∈ *I*(*T*), *e* ∈ *E*. These states (*t*_*j*_, *μ*^*t*_*j*_^, *ν*^*t*_*j*_^) ∈ *I*(*T*) exist in some accepted states. The extended transitional function *ϑ*^*∗*^ is defined as follows:

(1) $$\begin{array}{c} \vartheta^{*}\left(\left(t_{i},\mu^{t_{i}},\nu^{t_{i}}\right),e_{1}e_{2}\ldots e_{n}\right)=\left\{\begin{array}{cc} \left(t_{i},\mu^{t_{i}},\nu^{t_{i}}\right), & \text{if }n=0;\\ \left(\vartheta \left(\vartheta^{*}\left(t_{i},\mu^{t_{i}},\nu^{t_{i}}\right),e_{1}e_{2}\ldots e_{n-1}\right),e_{n}\right), & \text{if }n\neq 0, \end{array}\right. \end{array}$$

where *e*_1_*e*_2_ … *e*_*n*_ ∈ *E*^*∗*^ is the finite set of finite strings (words/sequences of input letters (symbols)) accepted by the automata.

**Example 1 .**

The following is considered:

1. *T*={*t*_1_, *t*_2_, *t*_3_}, the finite family of states.
2. *I*(*T*)={(*t*_*i*_, *μ*^*t*_*i*_^, *ν*^*t*_*i*_^) : *t*_*i*_ ∈ *T*, *μ* : *T*⟶(0,1], *ν* : *T*⟶[0,1) and 0 ≤ *μ*(*t*)+*ν*(*t*) ≤ 1}={(*t*_1_, 1,0), (*t*_2_, 0.4, 0.5), (*t*_3_, 0.3, 0.7)}, the finite family of states with *s*_*i*_=(*t*_1_, 1,0) as initial state.
3. *E*={*e*_1_, *e*_2_}, the collection of input letters/symbols.

The transitional mapping *ϑ* : *I*(*T*) × *E*⟶*I*(*T*) for the accepting states *t*_3_, *t*_2_ is defined as follows:

(2) $$\begin{array}{c} \vartheta \left(\left(t_{1},1,0\right),e_{1}\right)=\left(t_{1},1,0\right);\\ \vartheta \left(\left(t_{2},0.4,0.5\right),e_{1}\right)=\left(t_{1},1,0\right);\\ \vartheta \left(\left(t_{3},0.3,0.7\right),e_{1}\right)=\left(t_{2},0.4,0.5\right);\\ \vartheta \left(\left(t_{1},1,0\right),e_{2}\right)=\left(t_{3},0.3,0.7\right);\\ \vartheta \left(\left(t_{2},0.4,0.5\right),e_{2}\right)=\left(t_{3},0.3,0.7\right);\\ \vartheta \left(\left(t_{3},0.3,0.7\right),e_{2}\right)=\left(t_{3},0.3,0.7\right), \end{array}$$

with the transition diagram in Figure 2.

Then, *G*={(*t*_2_, 0.4, 0.5), (*t*_3_, 0.3, 0.7)} is an intuitionistic fuzzy set of accepting states. Thus, *AT*=(*T*, *I*(*T*), *ϑ*, *s*_*i*_, *E*, *G*). If we define mappings as follows:

(3) $$\begin{array}{c} f_{e_{1}}\left(t_{1},1,0\right)=\vartheta^{*}\left(\left(t_{1},1,0\right),e_{1}\right),\\ f_{e_{1}}\left(t_{2},0.4,0.5\right)=\vartheta^{*}\left(\left(t_{2},0.4,0.5\right),e_{1}\right),\\ f_{e_{1}}\left(t_{3},0.3,0.7\right)=\vartheta^{*}\left(\left(t_{3},0.3,0.7\right),e_{1}\right),\\ f_{e_{2}}\left(t_{1},1,0\right)=\vartheta^{*}\left(\left(t_{1},1,0\right),e_{2}\right),\\ f_{e_{2}}\left(t_{2},0.4,0.5\right)=\vartheta^{*}\left(\left(t_{2},0.4,0.5\right),e_{2}\right),\\ f_{e_{2}}\left(t_{3},0.3,0.7\right)=\vartheta^{*}\left(\left(t_{3},0.3,0.7\right),e_{2}\right),\\ f_{\wedge }\left(t_{i},\mu^{t_{i}},\nu^{t_{i}}\right)=\vartheta^{*}\left(\left(t_{i},\mu^{t_{i}},\nu^{t_{i}}\right),\wedge \right), \end{array}$$

where (*t*_*i*_, *μ*^*t*_*i*_^, *ν*^*t*_*i*_^) ∈ *I*(*T*) and ∧∈*E*^*∗*^(an empty sequence) make a table (see Table 1) for *f*_∧_, *f*_*e*_1__ and *f*_*e*_2__ that shows their effects on the states *t*_1_, *t*_2_ and *t*_3_.

We are now interested to determine whether *f*_∧_, *f*_*e*_1__ and *f*_*e*_2__ form a monoid under the composition of functions.

Elements *f*_*e*_1_*e*_1__, *f*_*e*_2_*e*_1__ of Table 2 do not exist in the set. Therefore, {*f*_∧_, *f*_*e*_1__, *f*_*e*_2__} is not a monoid. Now, it is expanded to {*f*_∧_, *f*_*e*_1__, *f*_*e*_2__, *f*_*e*_1_*e*_1__, *f*_*e*_2_*e*_1__} and this is established as monoid *M*_AT_, which corresponds to FDFIFA AT=(*T*, *I*(*T*), *ϑ*, *s*_*i*_, *E*, *G*).

## 3. Monoid of Fully Deterministic Finite-State Intuitionistic Fuzzy Automata

Let AT=(*T*, *I*(*T*), *ϑ*, *s*_*i*_, *E*, *G*) be an FDFIFA. For any input string or sequence *e*_1_*e*_2_ … *e*_*n*_ ∈ *E*^*∗*^, each state *t*_*i*_ ∈ *T* with membership *μ*^*t*_*i*_^ and nonmembership *ν*^*t*_*i*_^ is transited to another state (*t*_*j*_, *μ*^*t*_*j*_^, *ν*^*t*_*j*_^) ∈ *G*. If *f*_*e*_1_*e*_2_…*e*_*n*__ : *I*(*T*)⟶*I*(*T*) is defined as *f*_*e*_1_*e*_2_…*e*_*n*__(*t*_*i*_, *μ*^*t*_*i*_^, *ν*^*t*_*i*_^)=*ϑ*^*∗*^((*t*_*i*_, *μ*^*t*_*i*_^, *ν*^*t*_*i*_^), *e*_1_*e*_2_ … *e*_*n*_) for each *e*_1_*e*_2_ … *e*_*n*_ ∈ *E*^*∗*^ and (*t*_*i*_, *μ*^*t*_*i*_^, *ν*^*t*_*i*_^) ∈ *I*(*T*), then *M*_AT_={*f*_*e*_1_*e*_2_…*e*_*n*__ : *e*_1_*e*_2_ … *e*_*n*_ ∈ *E*^*∗*^} is a collection, which corresponds to FDFIFA AT. Clearly, ° is a binary operation on *M*_AT_ such that for any *f*_*e*_1_*e*_2_…*e*_*k*__, *f*_*e*_1_*e*_2_…*e*_*l*__ and *f*_*e*_1_*e*_2_…*e*_*m*__ ∈ *M*_AT_ with:

(4) $$\begin{array}{c} f_{e_{1}e_{2}\ldots e_{k}}\left(t_{i},\mu^{t_{i}},\nu^{t_{i}}\right)=\vartheta^{*}\left(\left(t_{i},\mu^{t_{i}},\nu^{t_{i}}\right),e_{1}e_{2}\ldots e_{k}\right),\\ f_{e_{1}e_{2}\ldots e_{l}}\left(t_{i},\mu^{t_{i}},\nu^{t_{i}}\right)=\vartheta^{*}\left(\left(t_{i},\mu^{t_{i}},\nu^{t_{i}}\right),e_{1}e_{2}\ldots e_{l}\right),\\ f_{e_{1}e_{2}\ldots e_{m}}\left(t_{i},\mu^{t_{i}},\nu^{t_{i}}\right)=\vartheta^{*}\left(\left(t_{i},\mu^{t_{i}},\nu^{t_{i}}\right),e_{1}e_{2}\ldots e_{k}\right), \end{array}$$

where (*t*_*i*_, *μ*^*t*_*i*_^, *ν*^*t*_*i*_^) ∈ *I*(*T*) and *k*, *l*, *m*=1,2,…*n* determine the length of string, *I*(*T*) is an intuitionistic fuzzy subset of states with grade of membership (HTML translation failed) and grade of nonmembership *ν* : *T*⟶[0,1), *E*^*∗*^ is the finite set of finite strings (words/sequences of input letters/symbols) accepted by the automata, and *ϑ*^*∗*^ is the extended transitional function. We have the following:

(5) $$\begin{array}{c} f_{e_{1}e_{2}\ldots e_{k}}{}^{\circ}\left(f_{e_{1}e_{2}\ldots e_{l}}{}^{\circ}f_{e_{1}e_{2}\ldots e_{m}}\right)=\left(f_{e_{1}e_{2}\ldots e_{k}}{}^{\circ}f_{e_{1}e_{2}\ldots e_{l}}\right){}^{\circ}f_{e_{1}e_{2}\ldots e_{m}}, \end{array}$$

which turns FDFIFA *M*_*AT*_ into monoid, called an FDFIFA monoid (under the composition of mappings). The expression *f*_*e*_1_*e*_2_…*e*_*k*__°*f*_*e*_1_*e*_2_…*e*_*l*__=*f*_*e*_1_*e*_2_…*e*_*k*_*e*_1_*e*_2_…*e*_*l*__ represents the overall state transition through *ϑ*^*∗*^ in the FDFIFA. FDFIFA contain a finite collection of states; thus, if the order of the collection of *I*(*T*) is *n*, that is, |*I*(*T*)|=*n*, then the monoid order is |*M*_AT_| ≤ *n*^*n*^.

**Definition 1 .**

Let (*M*_AT_,°) be an FDFIFA monoid corresponding to the automata AT, where:

(6) $$\begin{array}{c} \text{AT}=\left(T,I\left(T\right),\vartheta ,s_{i},E,G\right),\vartheta \left(\left(t_{i},\mu^{t_{i}},\nu^{t_{i}}\right),e\right)=\left(t_{j},\mu^{t_{j}},\nu^{t_{j}}\right). \end{array}$$

The extended transitional function *ϑ*^*∗*^ is defined as follows:

(7) $$\begin{array}{c} \vartheta^{*}\left(\left(t_{i},\mu^{t_{i}},\nu^{t_{i}}\right),e_{1}e_{2}\ldots e_{n}\right)=\left\{\begin{array}{cc} \left(t_{i},\mu^{t_{i}},\nu^{t_{i}}\right), & \text{if }n=0;\\ \left(\vartheta \left(\vartheta^{*}\left(t_{i},\mu^{t_{i}},\nu^{t_{i}}\right),e_{1}e_{2}\ldots e_{n-1}\right),e_{n}\right), & \text{if }n\neq 0. \end{array}\right. \end{array}$$

*M*_*AT*1_ is considered corresponding to the automata:

(8) $$\begin{array}{c} AT_{1}=\left(T_{1},I{\left(T\right)}_{1},\vartheta_{1},s_{i1},E_{1},G_{1}\right),\vartheta_{1}\left(\left(t_{i1},\mu^{t_{i1}},\nu^{t_{i1}}\right),\overset{´}{e}\right)=\left(t_{j1},\mu^{t_{j1}},\nu^{t_{j1}}\right). \end{array}$$

Then, *ϑ*_1_=*ϑ*/*I*(*P*)_1_ × *E*_1_, and

(9) $$\begin{array}{c} \vartheta_{1}^{*}=\frac{\vartheta^{*}}{I{\left(T\right)}_{1}}\times E_{1}^{*}, \end{array}$$

where (*t*_*i*_, *μ*^*t*_*i*_^, *ν*^*t*_*i*_^), (*t*_*j*_, *μ*^*t*_*j*_^, *ν*^*t*_*j*_^) ∈ *I*(*T*), *e* ∈ *E*, *e*_1_*e*_2_ … *e*_*n*_ ∈ *E*^*∗*^, $\left(t_{i1},\mu^{t_{i1}},\nu^{t_{i1}}\right),\left(t_{j1},\mu^{t_{j1}},\nu^{t_{j1}}\right)\in I{\left(T\right)}_{1},\overset{´}{e}\in E_{1}\subseteq E$, *T*_1_⊆*T*, *I*(*T*)_1_⊆*I*(*T*), \\*E*_1_^*∗*^⊆*E*^*∗*^, *s*_*i*_=*s*_*i*1_ and *G*_1_⊆*G*. If *M*_*AT*1_ is closed under the binary operation °, symbolically, *f*_*e*_1_*e*_2_…*e*_*k*__°*f*_*e*_1_*e*_2_…*e*_*l*__ ∈ *M*_*AT*1_∀ *f*_*e*_1_*e*_2_…*e*_*k*__, *f*_*e*_1_*e*_2_…*e*_*l*__ ∈ *M*_*AT*1_, then (*M*_*AT*1_,°) is known as a submonoid automaton of (*M*_*AT*_,°).

**Definition 2 .**

Any two FDFIFA monoids can be related to each other employing structure-preserving maps, commonly known as homomorphisms. Such maps not only preserve the binary operations used to design semigroups on FDFIFA but also the components involved in the formulation of FDFIFAs. Formally, if (*M*_*AT*_,°) and (*M*_*AT*1_, °_1_) are any two FDFIFA monoids, then a map *θ* : *M*_*AT*_⟶*M*_*AT*1_ defined as *θ*(*f*_*e*_1_*e*_2_…*e*_*n*__)=*f*_*ψ*(*e*_1_*e*_2_ … *e*_*n*_)_ is called an FDFIFA monoid homomorphism, and if *θ*(*f*_∧_)=*f*_*ψ*(∧)_=*f*_∧′_ and ∀*f*_*e*_1_*e*_2_…*e*_*k*__, *f*_*e*_1_*e*_2_…*e*_*l*__ ∈ *M*_*AT*_,

(10) $$\begin{array}{c} \theta \left(f_{e_{1}e_{2}\ldots e_{k}}{}^{\circ}f_{e_{1}e_{2}\ldots e_{l}}\right)=\theta \left(f_{e_{1}e_{2}\ldots e_{k}e_{1}e_{2}\ldots e_{l}}\right)\\ =f_{\psi \left(e_{1}e_{2}\ldots e_{k}e_{1}e_{2}\ldots e_{l}\right)}\\ =f_{\psi \left(e_{1}e_{2}\ldots e_{k}\right)\psi \left(e_{1}e_{2}\ldots e_{l}\right)}\\ =f_{\psi \left(e_{1}e_{2}\ldots e_{k}\right)}{{}^{\circ}}_{1}f_{\psi \left(e_{1}e_{2}\ldots e_{l}\right)}\\ =\theta \left(f_{e_{1}e_{2}\ldots e_{k}}\right){{}^{\circ}}_{1}\theta \left(f_{e_{1}e_{2}\ldots e_{l}}\right), \end{array}$$

where ′′∧′′(an empty sequence) ∈ *E*^*∗*^, ′′∧′′′(an empty sequence) ∈ *E*_1_^*∗*^, and *ψ* : *E*^*∗*^⟶*E*_1_^*∗*^ is a mapping, defined as ∀*e*_1_*e*_2_ … *e*_*k*_, *e*_1_*e*_2_ … *e*_*l*_ ∈ *E*^*∗*^, *ψ*(*e*_1_*e*_2_ … *e*_*k*_*e*_1_*e*_2_ … *e*_*l*_)=*ψ*(*e*_1_*e*_2_ … *e*_*k*_)*ψ*(*e*_1_*e*_2_ … *e*_*l*_). If *θ* is a homomorphism that also establishes a one-to-one correspondence between *M*_*AT*_ and *M*_*AT*1_, then it is termed to be an isomorphism and the FDFIFA monoids are denoted by *M*_*AT*_≃*M*_*AT*1_.

## 4. Intuitionistic Fuzzy Inference Rule on FDFIFA Monoid

On the semigroup of FDFIFA, intuitionistic fuzzy inference is a cognitive procedure that proceeds to a new decision or statement based on one or more previous decisions or propositions. In general, FDFIFA inference is divided into two components. The premise is a well-known decision used as a starting point for inference. The second is the conclusion, which is a fresh decision generated by the proposition. The following inference rules are offered based on the characteristics of homomorphic mapping:

  Premise 1: if *a* ∈ *X* semigroup, then *b* ∈ *Y* must be a semigroup.
  Premise 2: if $a\in \overset{´}{X}$ is a semigroup, then
  Conclusion: $b\in \overset{´}{Y}=\overset{´}{X}{}^{\circ}\left(X⟶Y\right)$, where ° is a binary operation and *X*⟶*Y* is a homomorphism.

The intuitionistic fuzzy inference system is made up of certain inference rules that must obey certain arithmetic requirements. The relationship between *X* and *Y* for Premise1 is *X*⟶*Y*, which is a homomorphism, grades of membership and nonmembership corresponding to an intuitionistic fuzzy relation matrix *F*, which is defined as follows:

(11) $$\begin{array}{c} F\left(p,q\right)=\left(\mu_{X⟶Y}\left(p,q\right),\nu_{X⟶Y}\left(p,q\right)\right)\\ =\left[\left(\mu_{X}\left(p\right)\wedge \mu_{Y}\left(q\right)\right)\vee \left(1-\mu_{X}\left(p\right)\right),\left(\nu_{X}\left(p\right)\vee \nu_{Y}\left(q\right)\right)\wedge \left(1-\nu_{X}\left(p\right)-\varepsilon \right)\right], \end{array}$$

where *μ*_*X*⟶*Y*_(*p*, *q*), *ν*_*X*⟶*Y*_(*p*, *q*) are the grades of membership and nonmembership for intuitionistic inference rule, *ϵ* is an error of hesitancy, *μ*_*Y*_(*q*), *ν*_*Y*_(*q*) are the grades of membership and nonmembership for the assumption that *q* ∈ *Y* is a semigroup, and *μ*_*X*_(*p*), *ν*_*X*_(*p*) are the grades of membership and nonmembership for the assumption that *p* ∈ *X* is a semigroup, and ∨ is an “or” operation and ∧ is an  “ and” operation:

(12) $$\begin{array}{c} \overset{´}{Y}=\overset{´}{X}{}^{\circ}\left(X⟶Y\right). \end{array}$$

The inference relationship between $\overset{´}{X}$ and *X* to *Y* can be used to synthesize the conclusion $\overset{´}{Y}$. *F* can be used to obtain the conclusion's membership and nonmembership functions:

(13) $$\begin{array}{c} \left(\mu_{\overset{´}{Y}}\left(q\right),\nu_{\overset{´}{Y}}\left(q\right)\right)=\left(\mu_{\overset{´}{X}}\left(p\right),\nu_{\overset{´}{X}}\left(p\right)\right){}^{\circ}F\left(p,q\right). \end{array}$$

The following is a description of °, the synthetic binary operator:

(14) $$\begin{array}{c} \left(\mu_{\overset{´}{Y}}\left(q\right),\nu_{\overset{´}{Y}}\left(q\right)\right)=\left(\mu_{\overset{´}{X}}\left(p\right),\nu_{\overset{´}{X}}\left(p\right)\right){}^{\circ}F\left(p,q\right)\\ =\left[\vee_{p\in X}\left\{\mu_{\overset{´}{X}}\left(p\right)\wedge \mu_{F}\left(p,q\right)\right\},\wedge_{p\in X}\left\{\nu_{\overset{´}{X}}\left(p\right)\vee \nu_{F}\left(p,q\right)\right\}\right], \end{array}$$

$\text{such that }0\leq \mu_{\overset{´}{Y}}\left(q\right)+\nu_{\overset{´}{Y}}\left(q\right)\leq 1$. In the classical fuzzy inference system, grade on membership of the fuzzy subset is a variable and variables are related through the operations defined on membership grades. However, in the inference system of FDFIFA semigroup, the FDFIFA semigroup serves as a variable and relationship between variables is exhibited using FDFIFA semigroup homomorphism.

## 5. Application

Automobiles provide millions around the world with a sense of freedom. People may now live, work, and engage in ways that were previously impossible a century ago. The automobile industry is the world's largest single most powerful economic driver. The earliest steam-powered vehicle was invented in 1672, and Nicolas-Joseph Cugnot created the first steam-powered automotive capable of human movement in 1770 [37], since then several automotive models are introduced with numerous modifications [38, 39]. The consumption of nonrenewable fuels, a major increase in the likelihood of unintentional fatality, the emission of noise and air  pollution, and the production of greenhouse gases are only a few of the present negative repercussions of widespread automobile use. The key benefit  of a hybrid automobile is  that it uses less gasoline and emits less CO_2_ [40] than a typical petrol or diesel-powered vehicle.

A hybrid vehicle is one that has multiple modes of propulsion, such as a gasoline or diesel engine and an electric motor. There are several kinds of hybrids, each of which functions differently [41]. Range extender hybrid automobiles (series hybrids) rely on their conventional engine to generate electricity to power a generator that recharges the batteries. Instead of propelling the car, the engine provides energy to the electric motor [42]. The well-known model is BMW i3 [43]. Plug-in hybrids are a kind of hybrid that can be recharged both at home and on the go, as the title indicates [44]. The BMW 330e, Mitsubishi Outlander, and Volvo V60 are just a few of the plug-in hybrids on the market. The hybrid car moves by combining at least one electrical motor with a gasoline engine, while the mechanism recovers energy through regenerative braking [45]. As result, lesser gasoline is burnt, resulting in higher fuel economy. Most of them use a high-voltage battery pack (different from the car's standard 12-volt battery) that is recharged by absorbing energy from deceleration that would otherwise be wasted to heat created by the brakes in traditional cars. (This is accomplished through the use of regenerative braking.)

The basic purpose of such regenerative braking is to transform kinetic energy (from the wheels) towards electrical energy and save it in batteries for future use in vehicle propulsion [46]. For reliable vehicle operation and control, these systems often use electric motors for both traction and regenerative braking. They also entail constant interactions between mechanical/electrical components and their controllers (electronic control units, ECUs). Faults in these technologies can have a substantial impact on the reliability and efficiency of automobile control and operation. According to the available literature, the focus of hybrid electric vehicle (HEV) studies has been on design and control methods for enhanced energy regeneration [47], best possible braking strategies [48], and mechanism level control to improve energy/fuel efficiency [49–51], with fault analysis receiving far less attention. A fault-tolerant power train topology for series hybrid electric vehicles was discussed by Song and Wang [52]. They looked at short-switch and open-switch failures that threaten motor drive unit reliability. Parsa and Toliyat [53] suggested a fault-tolerant control approach for five-phase permanent magnet motors. It was determined that the system could function securely with up to two phases lost without the need of any extra equipment. A basic on-board fault detection technique built on reference frame theory for detecting electric motor defects in HEVs at start-up and idle circumstances is described in [54]. Rothenhagen and Fuchs [55] present a spectator residual generation technique to identify current sensor problems.

In cascaded multiple converter devices, Jayabalan and Fahimi [56] proposed using statistical moments of higher powers to identify open-circuit and short-circuit failures. Merzouki et al. [57] discussed a parity relation-based residual generation technique for detecting and isolating actuator faults in electric vehicles. Existing HEV failure diagnostic methods are component-centric and may not explicitly incorporate communication or scheme interactions. This research looks at hardware, programming, and communication defects in HEV's regenerative braking (RBS) and proposes a data-driven technique for detecting and identifying them. Parametric and sensor-related problems (underlying physical faults), software logic faults, and interprocess communication defects (missed messages, several messages, and obsolete message faults) are among the defects investigated. The use of a series-parallel power train with regenerative braking is contemplated. The automobile is normally propelled by two power sources: (i) an internal combustion engine (ICE) and an electric generator; and (ii) an electric motor having a battery as the power storage system [58]. The various constituent components of the drive train design (with a series-parallel power train configuration) are shown in Figure 3. The car operates in an electricity-only mode when the speed or power demand is minimal (series mode). When the car's power requirement at the wheels is larger, the engine and the motor work together to push the vehicle forward (parallel mode). Ehsani et al. [59] provided further information about different drive train layouts. As a result, defining nominal and problematic behaviour, as well as developing detection and inference algorithms for rapid fault diagnosis, is crucial.

### 5.1. FDFIFA Monoid

Now, we construct an FDFIFA semigroup (*M*_*AT*_,°) fault diagnosis model for the hybrid electric vehicle regenerative braking system. Let (*M*_*AT*_,°) be an FDFIFA semigroup corresponding to the automata *AT*=(*T*, *I*(*T*), *ϑ*, *s*_*i*_, *E*, *G*), where *T* is a collection of states that the hybrid electric vehicle regenerative braking system can be in, such as normal, medium, or serious faults; *I*(*T*) is an intuitionistic fuzzy subset of states *T* with grade of membership *μ* : *T*⟶(0,1] and grade of nonmembership *ν* : *T*⟶[0,1); *E* is an input character signal set; *s*_*i*_ ∈ *I*(*T*) is the initial state of the processing signal; *G* is a fault state set and a subset of *I*(*T*); and *ϑ* : *I*(*T*) × *E*⟶*I*(*T*) is the transitional mapping with *ϑ*((*t*_*i*_, *μ*^*t*_*i*_^, *ν*^*t*_*i*_^), *e*)=(*t*_*j*_, *μ*^*t*_*j*_^, *ν*^*t*_*j*_^), where (*t*_*i*_, *μ*^*t*_*i*_^, *ν*^*t*_*i*_^), (*t*_*j*_, *μ*^*t*_*j*_^, *ν*^*t*_*j*_^) ∈ *I*(*T*), *e* ∈ *E*. These states (*t*_*j*_, *μ*^*t*_*j*_^, *ν*^*t*_*j*_^) ∈ *I*(*T*) exist in some accepted states. The extended transitional function *ϑ*^*∗*^ is defined as follows:

(15) $$\begin{array}{c} \vartheta^{*}\left(\left(t_{i},\mu^{t_{i}},\nu^{t_{i}}\right),e_{1}e_{2}\ldots e_{n}\right)=\left\{\begin{array}{cc} \left(t_{i},\mu^{t_{i}},\nu^{t_{i}}\right), & \text{if }n=0;\\ \left(\vartheta \left(\vartheta^{*}\left(t_{i},\mu^{t_{i}},\nu^{t_{i}}\right),e_{1}e_{2}\ldots e_{n-1}\right),e_{n}\right), & \text{if }n\neq 0, \end{array}\right. \end{array}$$

where *e*_1_*e*_2_ … *e*_*n*_ ∈ *E*^*∗*^ is the finite set of finite strings (words/sequences of input letters (symbols)) accepted by the automata. Because *s*_*i*_ ∈ *I*(*T*), *I*(*T*) denotes the entire states, *G*⊆*I*(*T*), and *ϑ* is a transition procedure from one state to another. The degree of FDFIFA semigroup membership and nonmembership can show the regenerative braking's degree of fault and accuracy. As a result, the degree of membership is utilized to indicate the severity of the defect. *G* and *E* are mostly treated in the following order:

(i) Fault state or output variable set **G**: the normal working condition represented by *W*_1_, battery current sensor fault represented by *W*_2_, battery temperature sensor fault denoted by *W*_3_, engine speed sensor fault denoted by *W*_4_, motor 1 current sensor fault denoted by *W*_5_, motor 1 speed sensor fault denoted by *W*_6_, vehicle speed sensor fault denoted by *W*_7_, wheel inertia fault denoted by *W*_8_, engine message loss fault denoted by *W*_9_, burst loss of engine message denoted by *W*_10_, burst loss of message from PTC denoted by *W*_11_, too many messages from battery denoted by *W*_12_, battery initial SOC fault denoted by *W*_13_, wheel radius fault denoted by *W*_14_, engine message faulty data denoted by *W*_15_, motor 1 message faulty data denoted by *W*_16_, and wheel message faulty data denoted by *W*_17_. The range of values from *W*_1_ to *W*_17_ is included inside the [0,1] interval. 0 in the interval denotes the absence of such a flaw. 1 denotes a major flaw [60].
(ii) Processing signal or input variable set **E**: the following 25 felt parameters are chosen as input variables: *e*_1_: battery SOC, *e*_2_: motor 2 torque demand, *e*_3_: wheel torque demand, *e*_4_: motor 1 torque demand, *e*_5_: engine torque demand, *e*_6_: battery temperature, *e*_7_: battery current, *e*_8_: driver torque demand, *e*_9_: motor 1 command, *e*_10_: gearbox speed, *e*_11_: wheel input speed, *e*_12_: wheel output speed, *e*_13_: wheel torque, *e*_14_: vehicle linear speed, *e*_15_: motor 1 speed, *e*_16_: motor 1 current, *e*_17_: clutch input speed, *e*_18_: engine command, *e*_19_: motor 2 command, *e*_20_: motor 2 speed, *e*_21_: motor 2 current, *e*_22_: engine speed, *e*_23_: clutch output speed, *e*_24_: mechanical accessory torque, and *e*_25_: wheel command [60].
(iii) The degrees to which each fault and accuracy parameter corresponds to the categories of “normal,” “serious,” and “medium” are presented in terms of membership and the intuitionistic degree of nonmembership grades as follows:
  (16) $$\begin{array}{c} \left(\mu_{\text{normal}},\nu_{\text{normal}}\right)=\left(\begin{array}{c} \left(1,0\right)\left(0.2,0.6\right)\left(0.1,0.8\right)\left(0.2,0.5\right)\left(0.1,0.8\right)\\ \left(0,0.9\right)\left(0,0.8\right)\left(0.1,0.6\right)\left(0.1,0.7\right)\\ \left(0,0.4\right)\left(0.2,0.6\right)\left(0.1,0.8\right)\left(0,0.9\right)\left(0.2,0.6\right)\left(0.2,0.7\right)\left(0,0.9\right)\left(0.1,0.8\right) \end{array}\right), \end{array}$$
  (17) $$\begin{array}{c} \left(\mu_{\text{serious}},\nu_{\text{serious}}\right)=\left(\begin{array}{c} \left(0,0.6\right)\left(0.2,0.7\right)\left(0.3,0.7\right)\left(0.4,0.5\right)\left(0.6,0.2\right)\left(0.8,0.1\right)\left(0.6,0.3\right)\\ \left(0.7,0.2\right)\left(0.1,0.7\right)\left(0.3,0.6\right)\\ \left(0.6,0.4\right)\left(0.2,0.8\right)\left(0.1,0.9\right)\left(0.7,0.2\right)\left(0.3,0.7\right)\left(0.1,0.9\right)\left(0.2,0.8\right) \end{array}\right), \end{array}$$
  (18) $$\begin{array}{c} \left(\mu_{\text{medium}},\nu_{\text{medium}}\right)=\left(\begin{array}{c} \left(1,0\right)\left(0.3,0.4\right)\left(0.2,0.8\right)\left(0.1,0.9\right)\left(0.4,0.3\right)\left(0.3,0.4\right)\left(0.3,0.7\right)\\ \left(0.2,0.7\right)\left(0.1,0.8\right)\left(0,0.6\right)\left(0,0.9\right)\left(0.5,0.4\right)\\ \left(0.2,0.7\right)\left(0.3,0.2\right)\left(0.4,0.6\right)\left(0.2,0.5\right)\left(0.4,0.5\right) \end{array}\right). \end{array}$$

### 5.2. Intuitionistic Fuzzy Inference Model

Faults are divided into three categories to make diagnosis easier: serious fault, medium fault, and no fault. The result is processed as follows, based on the output state of the intuitionistic fuzzy inference model of FDFIFA semigroup:

If 0.60 ≤ *μ*(*W*_*i*_) ≤ 1 and 0 ≤ *ν*(*W*_*i*_) ≤ 0.40, *W*_*i*_ is level 1, recognized as the serious fault.

When 0.25 < *μ*(*W*_*i*_) < 0.60 and 0.40 < *ν*(*W*_*i*_) < 0.75, *W*_*i*_ is level 2, recognized as the medium defect.

If *μ*(*W*_*i*_) ≤ 0.25 and *ν*(*W*_*i*_) ≤ 0.75, *W*_*i*_ is normal, recognized as no fault.

The seriousness of the defect can be obtained by utilizing this information. The FDFIFA semigroup's inference system has now been completely specified, comprising variables, membership functions, nonmembership functions, and the essential rules for diagnosing faults. The FDIFA semigroup rule viewer permits us to totally comprehend the entire intuitionistic fuzzy inference process at once. It also demonstrates the influences of the membership and nonmembership functions on the overall outcomes of the intuitionistic fuzzy inference. Our prior work has a full description of how to design an intuitionist fuzzy inference system for fault detection [24]. If the problem being examined is complex in nature subject to several conflicting factors, then FDFIFA semigroup inference is an appropriate tool for its solution. Semigroup's intuitionistic fuzzy inference model is put to the test with a collection of real data to see whether it can correctly identify a hybrid electric vehicle regenerative braking system issue. The intuitionistic fuzzy inference model can be employed if the fault can be appropriately diagnosed. The corresponding parameters are monitored and their values are acquired when *W*_5_, *W*_6_, *W*_7_, and *W*_8_ are defective. The data are utilized as input vectors in simulation functions to compute the output of an intuitionistic fuzzy inference model. The fault criterion is used to determine whether or not a flaw exists. The test result shows that 5, 6, and 12 in *W*_*i*_ − *out* signify distinct types of faults illustrated as follows:

(19) $$\begin{array}{c} \text{Input vector}=\left(\begin{array}{c} \left(0.2,0.7\right)\left(0.1,0.7\right)\left(0.2,0.7\right)\left(0.6,0.3\right)\left(0,0.8\right)\\ \left(0,0.9\right)\left(0.1,0.7\right)\left(0.1,0.8\right)\left(0,0.9\right)\left(0.1,0.7\right)\left(0.2,0.7\right)\\ \left(0,0.8\right)\left(0,0.9\right)\left(0.1,0.7\right)\left(0.1,0.8\right)\left(0,0.9\right) \end{array}\right),\\ \text{Cause of fault}=W_{5}\text{ serious fault,}\\ \text{Input vector}=\left(\begin{array}{c} \left(0.2,0.6\right)\left(0.1,0.7\right)\left(0.2,0.6\right)\left(0.1,0.8\right)\left(0.4,0.5\right)\\ \left(0,0.8\right)\left(0.1,0.7\right)\left(0.1,0.8\right)\left(0,0.9\right)\left(0.2,0.6\right)\left(0.1,0.7\right)\\ \left(0.2,0.6\right)\left(0.1,0.7\right)\left(0.2,0.6\right)\left(0.1,0.7\right)\left(0.2,0.6\right) \end{array}\right),\\ \text{Cause of fault}=W_{6}\text{ medium fault,}\\ \text{Input vector}=\left(\begin{array}{c} \left(0.2,0.6\right)\left(0.1,0.8\right)\left(0.2,0.6\right)\left(0.1,0.7\right)\left(0.2,0.6\right)\\ \left(0.1,0.7\right)\left(0.2,0.6\right)\left(0.2,0.7\right)\left(0.1,0.8\right)\left(0,0.8\right)\left(0.6,0.3\right)\\ \left(0.1,0.8\right)\left(0.1,0.7\right)\left(0,0.8\right)\left(0.1,0.8\right)\left(0.1,0.7\right) \end{array}\right),\\ \text{Cause of fault}=W_{12}\text{ serious fault.} \end{array}$$

Suppose (*M*_*AT*1_, °_1_) be an FDFIFA semigroup corresponding to the automata *AT*1, (*M*_*AT*2_, °_2_) be an FDFIFA semigroup corresponding to the automata *AT*2 as constructed above, and *θ* : *M*_*AT*1_⟶*M*_*AT*2_ is an inference rule in terms of FDFIFA homomorphism. In the aforesaid application, the inference model for fault diagnostics can be built as follows:

  Premise 1: if *M*_*AT*1_ parameter *a* is normal, *M*_*AT*2_ output *b* is serious.
  Premise 2: if *M*_*AT*1_ parameter $\overset{´}{a}$ is medium, then
  Conclusion: try to figure out what the fault level of the output $\overset{´}{b}$ in *M*_*AT*2_.

The degree of membership and nonmembership that corresponds to each inference step of the model can be determined using the intuitionistic fuzzy inference system, starting with the known condition.

Step 1: the intuitionistic fuzzy relation matrix *F* can be calculated using Premise 1 and the formula (11), as well as the intuitionistic fuzzy degree of membership and nonmembership given by the aforementioned expressions (16) and (17).
  (20) $$\begin{array}{c} F\left(a,b\right)=\left(\mu_{M_{AT1}⟶M_{AT2}}\left(a,b\right),\nu_{M_{AT1}⟶M_{AT2}}\left(a,b\right)\right)\\ =\left[\begin{array}{c} \left(\mu_{M_{AT1}}\left(a\right)\wedge \mu_{M_{AT2}}\left(b\right)\right)\vee \left(1-\mu_{M_{AT1}}\left(a\right)\right)\\ \left(\nu_{M_{AT1}}\left(a\right)\vee \nu_{M_{AT2}}\left(b\right)\right)\wedge \left(1-\nu_{M_{AT1}}\left(a\right)-\varepsilon \right) \end{array}\right],\\ A=\left(\left(\mu_{M_{AT1}}\left(a\right),\nu_{M_{AT1}}\left(a\right)\right)\left(\wedge ,\vee \right)\left(\mu_{M_{AT2}}\left(b\right),\nu_{M_{AT2}}\left(b\right)\right)\right)\\ =\left[\begin{array}{ccccccccccccccccc} \left(0,0.6\right) & \left(0.2,0.7\right) & \left(0.3,0.7\right) & \left(0.4,0.5\right) & \left(0.6,0.2\right) & \left(0.8,0.1\right) & \left(0.6,0.3\right) & \left(0.7,0.2\right) & \left(0.1,0.7\right) & \left(0.3,0.6\right) & \left(0.6,0.4\right) & \left(0.2,0.8\right) & \left(0.1,0.9\right) & \left(0.7,0.2\right) & \left(0.3,0.7\right) & \left(0.1,0.9\right) & \left(0.2,0.8\right)\\ \left(0,0.6\right) & \left(\text{0.}2\text{,0.}7\right) & \left(\text{0.}2\text{,0.}7\right) & \left(\text{0.}2\text{,0.}6\right) & \left(\text{0.}2\text{,0.}6\right) & \left(\text{0.}2\text{,0.}6\right) & \left(\text{0.}2\text{,0.}6\right) & \left(\text{0.}2\text{,0.}6\right) & \left(\text{0.}1\text{,0.}7\right) & \left(\text{0.}2\text{,0.}6\right) & \left(\text{0.}2\text{,0.}6\right) & \text{0.}2\text{,0.}8 & \left(0.1,0.9\right) & \left(\text{0.}2\text{,0.}6\right) & \left(\text{0.}2\text{,0.}7\right) & \left(0.1,0.9\right) & \left(0.2,0.8\right)\\ \left(\text{0,0.}8\right) & \left(\text{0.}1\text{,0.}8\right) & \left(\text{0.}1\text{,0.}8\right) & \left(\text{0.}1\text{,0.}8\right) & \left(\text{0.}1\text{,0.}8\right) & \left(\text{0.}1\text{,0.}8\right) & \left(\text{0.}1\text{,0.}8\right) & \left(\text{0.}1\text{,0.}8\right) & \left(\text{0.}1\text{,0.}8\right) & \left(\text{0.}1\text{,0.}8\right) & \left(\text{0.}1\text{,0.}8\right) & \left(\text{0.}1\text{,0.}8\right) & \left(0.1,0.9\right) & \left(\text{0.}1\text{,0.}8\right) & \left(\text{0.}1\text{,0.}8\right) & \left(0.1,0.9\right) & \left(\text{0.}1\text{,0.}8\right)\\ \left(0,0.6\right) & \left(\text{0.}2\text{,0.}7\right) & \left(\text{0.}2\text{,0.}7\right) & \left(\text{0.}2\text{,0.}5\right) & \left(\text{0.}2\text{,0.}5\right) & \left(\text{0.}2\text{,0.}5\right) & \left(\text{0.}2\text{,0.}5\right) & \left(\text{0.}2\text{,0.}5\right) & \left(\text{0.}2\text{,0.}5\right) & \left(\text{0.}2\text{,0.}5\right) & \left(\text{0.}2\text{,0.}6\right) & \left(\text{0.}2\text{,0.}8\right) & \left(0.1,0.9\right) & \left(\text{0.}2\text{,0.}5\right) & \left(\text{0.}2\text{,0.}7\right) & \left(0.1,0.9\right) & \left(\text{0.}2\text{,0.}8\right)\\ \left(\text{0,0.}8\right) & \left(\text{0.}1\text{,0.}8\right) & \left(\text{0.}1\text{,0.}8\right) & \left(\text{0.}1\text{,0.}8\right) & \left(\text{0.}1\text{,0.}8\right) & \left(\text{0.}1\text{,0.}8\right) & \left(\text{0.}1\text{,0.}8\right) & \left(\text{0.}1\text{,0.}8\right) & \left(\text{0.}1\text{,0.}8\right) & \left(\text{0.}1\text{,0.}8\right) & \left(\text{0.}1\text{,0.}8\right) & \left(\text{0.}1\text{,0.}8\right) & \left(0.1,0.9\right) & \left(\text{0.}1\text{,0.}8\right) & \left(\text{0.}1\text{,0.}8\right) & \left(0.1,0.9\right) & \left(\text{0.}1\text{,0.}8\right)\\ \left(\text{0,0.}9\right) & \left(\text{0,0.}9\right) & \left(\text{0,0.}9\right) & \left(\text{0,0.}9\right) & \left(\text{0,0.}9\right) & \left(\text{0,0.}9\right) & \left(\text{0,0.}9\right) & \left(\text{0,0.}9\right) & \left(\text{0,0.}9\right) & \left(\text{0,0.}9\right) & \left(\text{0,0.}9\right) & \left(\text{0,0.}9\right) & \left(\text{0,0.}9\right) & \left(\text{0,0.}9\right) & \left(\text{0,0.}9\right) & \left(\text{0,0.}9\right) & \left(\text{0,0.}9\right)\\ \left(\text{0,0.}8\right) & \left(\text{0,0.}8\right) & \left(\text{0,0.}8\right) & \left(\text{0,0.}8\right) & \left(\text{0,0.}8\right) & \left(\text{0,0.}8\right) & \left(\text{0,0.}8\right) & \left(\text{0,0.}8\right) & \left(\text{0,0.}8\right) & \left(\text{0,0.}8\right) & \left(\text{0,0.}8\right) & \left(\text{0,0.}8\right) & \left(\text{0,0.}9\right) & \left(\text{0,0.}8\right) & \left(\text{0,0.}8\right) & \left(\text{0,0.}9\right) & \left(\text{0,0.}8\right)\\ \left(\text{0,0.}6\right) & \left(\text{0.}1\text{,0.}7\right) & \left(\text{0.}1\text{,0.}7\right) & \left(\text{0.}1\text{,0.}6\right) & \left(\text{0.}1\text{,0.}6\right) & \left(\text{0.}1\text{,0.}6\right) & \left(\text{0.}1\text{,0.}6\right) & \left(\text{0.}1\text{,0.}6\right) & \left(\text{0.}1\text{,0.}7\right) & \left(\text{0.}1\text{,0.}6\right) & \left(\text{0.}1\text{,0.}6\right) & \left(\text{0.}1\text{,0.}8\right) & \left(\text{0.}1\text{,0.}9\right) & \left(\text{0.}1\text{,0.}6\right) & \left(\text{0.}1\text{,0.}7\right) & \left(\text{0.}1\text{,0.}9\right) & \left(\text{0.}1\text{,0.}8\right)\\ \left(\text{0,0.}7\right) & \left(\text{0.}1\text{,0.}7\right) & \left(\text{0.}1\text{,0.}7\right) & \left(\text{0.}1\text{,0.}7\right) & \left(\text{0.}1\text{,0.}7\right) & \left(\text{0.}1\text{,0.}7\right) & \left(\text{0.}1\text{,0.}7\right) & \left(\text{0.}1\text{,0.}7\right) & \left(\text{0.}1\text{,0.}7\right) & \left(\text{0.}1\text{,0.}7\right) & \left(\text{0.}1\text{,0.}7\right) & \left(\text{0.}1\text{,0.}8\right) & \left(\text{0.}1\text{,0.}9\right) & \left(\text{0.}1\text{,0.}7\right) & \left(\text{0.}1\text{,0.}7\right) & \left(\text{0.}1\text{,0.}9\right) & \left(\text{0.}1\text{,0.}8\right)\\ \left(\text{0,0.}6\right) & \left(\text{0,0.}7\right) & \left(\text{0,0.}7\right) & \left(\text{0,0.}5\right) & \left(\text{0,0.}4\right) & \left(\text{0,0.}4\right) & \left(\text{0,0.}4\right) & \left(\text{0,0.}4\right) & \left(\text{0,0.}7\right) & \left(\text{0,0.}6\right) & \left(\text{0,0.}4\right) & \left(\text{0,0.}8\right) & \left(\text{0,0.}9\right) & \left(\text{0,0.}4\right) & \left(\text{0,0.}7\right) & \left(\text{0,0.}9\right) & \left(\text{0,0.}8\right)\\ \left(\text{0,0.}6\right) & \left(\text{0.}2\text{,0.}7\right) & \left(\text{0.}2\text{,0.}7\right) & \left(\text{0.}2\text{,0.}6\right) & \left(\text{0.}2\text{,0.}6\right) & \left(\text{0.}2\text{,0.}6\right) & \left(\text{0.}2\text{,0.}6\right) & \left(\text{0.}2\text{,0.}6\right) & \left(\text{0.}1\text{,0.}7\right) & \left(\text{0.}2\text{,0.}6\right) & \left(\text{0.}2\text{,0.}6\right) & \left(\text{0.}2\text{,0.}8\right) & \left(\text{0.}1\text{,0.}9\right) & \left(\text{0.}2\text{,0.}6\right) & \left(\text{0.}2\text{,0.}7\right) & \left(\text{0.}1\text{,0.}9\right) & \left(\text{0.}2\text{,0.}8\right)\\ \left(\text{0,0.}8\right) & \left(\text{0.}1\text{,0.}8\right) & \left(\text{0.}1\text{,0.}8\right) & \left(\text{0.}1\text{,0.}8\right) & \left(\text{0.}1\text{,0.}8\right) & \left(\text{0.}1\text{,0.}8\right) & \left(\text{0.}1\text{,0.}8\right) & \left(\text{0.}1\text{,0.}8\right) & \left(\text{0.}1\text{,0.}8\right) & \left(\text{0.}1\text{,0.}8\right) & \left(\text{0.}1\text{,0.}8\right) & \left(\text{0.}1\text{,0.}8\right) & \left(\text{0.}1\text{,0.}9\right) & \left(\text{0.}1\text{,0.}8\right) & \left(\text{0.}1\text{,0.}8\right) & \left(\text{0.}1\text{,0.}9\right) & \left(\text{0.}1\text{,0.}8\right)\\ \left(\text{0,0.}9\right) & \left(\text{0,0.}9\right) & \left(\text{0,0.}9\right) & \left(\text{0,0.}9\right) & \left(\text{0,0.}9\right) & \left(\text{0,0.}9\right) & \left(\text{0,0.}9\right) & \left(\text{0,0.}9\right) & \left(\text{0,0.}9\right) & \left(\text{0,0.}9\right) & \left(\text{0,0.}9\right) & \left(\text{0,0.}9\right) & \left(\text{0,0.}9\right) & \left(\text{0,0.}9\right) & \left(\text{0,0.}9\right) & \left(\text{0,0.}9\right) & \left(\text{0,0.}9\right)\\ \left(\text{0,0.}6\right) & \left(\text{0.}2\text{,0.}7\right) & \left(\text{0.}2\text{,0.}7\right) & \left(\text{0.}2\text{,0.}6\right) & \left(\text{0.}2\text{,0.}6\right) & \left(\text{0.}2\text{,0.}6\right) & \left(\text{0.}2\text{,0.}6\right) & \left(\text{0.}2\text{,0.}6\right) & \left(\text{0.}1\text{,0.}7\right) & \left(\text{0.}2\text{,0.}6\right) & \left(\text{0.}2\text{,0.}6\right) & \left(\text{0.}2\text{,0.}8\right) & \left(\text{0.}1\text{,0.}9\right) & \left(\text{0.}2\text{,0.}6\right) & \left(\text{0.}2\text{,0.}7\right) & \left(\text{0.}1\text{,0.}9\right) & \left(\text{0.}2\text{,0.}8\right)\\ \left(\text{0,0.}7\right) & \left(\text{0.}2\text{,0.}7\right) & \left(\text{0.}2\text{,0.}7\right) & \left(\text{0.}2\text{,0.}7\right) & \left(\text{0.}2\text{,0.}7\right) & \left(\text{0.}2\text{,0.}7\right) & \left(\text{0.}2\text{,0.}7\right) & \left(\text{0.}2\text{,0.}7\right) & \left(\text{0.}1\text{,0.}7\right) & \left(\text{0.}2\text{,0.}7\right) & \left(\text{0.}2\text{,0.}7\right) & \left(\text{0.}2\text{,0.}8\right) & \left(\text{0.}1\text{,0.}9\right) & \left(\text{0.}2\text{,0.}7\right) & \left(\text{0.}2\text{,0.}7\right) & \left(\text{0.}1\text{,0.}9\right) & \left(\text{0.}2\text{,0.}8\right)\\ \left(\text{0,0.}9\right) & \left(\text{0,0.}9\right) & \left(\text{0,0.}9\right) & \left(\text{0,0.}9\right) & \left(\text{0,0.}9\right) & \left(\text{0,0.}9\right) & \left(\text{0,0.}9\right) & \left(\text{0,0.}9\right) & \left(\text{0,0.}9\right) & \left(\text{0,0.}9\right) & \left(\text{0,0.}9\right) & \left(\text{0,0.}9\right) & \left(\text{0,0.}9\right) & \left(\text{0,0.}9\right) & \left(\text{0,0.}9\right) & \left(\text{0,0.}9\right) & \left(\text{0,0.}9\right)\\ \left(\text{0,0.}8\right) & \left(\text{0.}1\text{,0.}8\right) & \left(\text{0.}1\text{,0.}8\right) & \left(\text{0.}1\text{,0.}8\right) & \left(\text{0.}1\text{,0.}8\right) & \left(\text{0.}1\text{,0.}8\right) & \left(\text{0.}1\text{,0.}8\right) & \left(\text{0.}1\text{,0.}8\right) & \left(\text{0.}1\text{,0.}8\right) & \left(\text{0.}1\text{,0.}8\right) & \left(\text{0.}1\text{,0.}8\right) & \left(\text{0.}1\text{,0.}8\right) & \left(\text{0.}1\text{,0.}9\right) & \left(\text{0.}1\text{,0.}8\right) & \left(\text{0.}1\text{,0.}8\right) & \left(\text{0.}1\text{,0.}9\right) & \left(\text{0.}1\text{,0.}9\right) \end{array}\right]\\ B=\left(\left(1-\mu_{M_{AT1}}\left(a\right)\right),\left(1-\nu_{M_{AT1}}\left(a\right)-\varepsilon \left(=0.1\right)\right)\right)\\ =\left(\begin{array}{c} \left(0,0.9\right)\left(0.8,0.3\right)\left(0.9,0.1\right)\left(0.8,0.4\right)\left(0.9,0.1\right)\\ \left(1,0\right)\left(1,0.1\right)\left(0.9,0.3\right)\left(0.9,0.2\right)\left(1,0.5\right)\\ \left(0.8,0.3\right)\left(0.9,0.1\right)\left(1,0\right)\left(0.8,0.3\right)\left(0.8,0.2\right)\left(1,0\right)\left(0.9,0.1\right) \end{array}\right)\\ F\left(a,b\right)=F_{\left(\mu ,\nu \right)}\left(a,b\right)=A\left(\vee ,\wedge \right)B\\ =\left[\begin{array}{ccccccccccccccccc} \left(\text{0,0.}6\right) & \left(\text{0.}2\text{,0.}7\right) & \left(\text{0.}3\text{,0.}7\right) & \left(\text{0.}4\text{,0.}7\right) & \left(\text{0.}6\text{,0.}2\right) & \left(\text{0.}8\text{,0.}1\right) & \left(\text{0.}6\text{,0.}3\right) & \left(\text{0.}7\text{,0.}2\right) & \left(\text{0.}1\text{,0.}7\right) & \left(\text{0.}3\text{,0.}6\right) & \left(\text{0.}6\text{,0.}4\right) & \left(\text{0.}2\text{,0.}8\right) & \left(\text{0.}1\text{,0.}9\right) & \left(\text{0.}7\text{,0.}2\right) & \left(\text{0.}3\text{,0.}7\right) & \left(\text{0.}1\text{,0.}9\right) & \left(\text{0.}2\text{,0.}8\right)\\ \left(\text{0.}8\text{,0.}3\right) & \left(\text{0.}8\text{,0.}3\right) & \left(\text{0.}8\text{,0.}3\right) & \left(\text{0.}8\text{,0.}3\right) & \left(\text{0.}8\text{,0.}3\right) & \left(\text{0.}8\text{,0.}3\right) & \left(\text{0.}8\text{,0.}3\right) & \left(\text{0.}8\text{,0.}3\right) & \left(\text{0.}8\text{,0.}3\right) & \left(\text{0.}8\text{,0.}3\right) & \left(\text{0.}8\text{,0.}3\right) & \left(\text{0.}8\text{,0.}3\right) & \left(\text{0.}8\text{,0.}3\right) & \left(\text{0.}8\text{,0.}3\right) & \left(\text{0.}8\text{,0.}3\right) & \left(\text{0.}8\text{,0.}3\right) & \left(\text{0.}8\text{,0.}3\right)\\ \left(\text{0.}9\text{,0.}1\right) & \left(\text{0.}9\text{,0.}1\right) & \left(\text{0.}9\text{,0.}1\right) & \left(\text{0.}9\text{,0.}1\right) & \left(\text{0.}9\text{,0.}1\right) & \left(\text{0.}9\text{,0.}1\right) & \left(\text{0.}9\text{,0.}1\right) & \left(\text{0.}9\text{,0.}1\right) & \left(\text{0.}9\text{,0.}1\right) & \left(\text{0.}9\text{,0.}1\right) & \left(\text{0.}9\text{,0.}1\right) & \left(\text{0.}9\text{,0.}1\right) & \left(\text{0.}9\text{,0.}1\right) & \left(\text{0.}9\text{,0.}1\right) & \left(\text{0.}9\text{,0.}1\right) & \left(\text{0.}9\text{,0.}1\right) & \left(\text{0.}9\text{,0.}1\right)\\ \left(\text{0.}8\text{, 0.}4\right) & \left(\text{0.}8\text{, 0.}4\right) & \left(\text{0.}8\text{, 0.}4\right) & \left(\text{0.}8\text{, 0.}4\right) & \left(\text{0.}8\text{, 0.}4\right) & \left(\text{0.}8\text{, 0.}4\right) & \left(\text{0.}8\text{, 0.}4\right) & \left(\text{0.}8\text{, 0.}4\right) & \left(\text{0.}8\text{, 0.}4\right) & \left(\text{0.}8\text{, 0.}4\right) & \left(\text{0.}8\text{, 0.}4\right) & \left(\text{0.}8\text{, 0.}4\right) & \left(\text{0.}8\text{, 0.}4\right) & \left(\text{0.}8\text{, 0.}4\right) & \left(\text{0.}8\text{, 0.}4\right) & \left(\text{0.}8\text{, 0.}4\right) & \left(\text{0.}8\text{, 0.}4\right)\\ \left(\text{0.}9\text{,0.}1\right) & \left(\text{0.}9\text{,0.}1\right) & \left(\text{0.}9\text{,0.}1\right) & \left(\text{0.}9\text{,0.}1\right) & \left(\text{0.}9\text{,0.}1\right) & \left(\text{0.}9\text{,0.}1\right) & \left(\text{0.}9\text{,0.}1\right) & \left(\text{0.}9\text{,0.}1\right) & \left(\text{0.}9\text{,0.}1\right) & \left(\text{0.}9\text{,0.}1\right) & \left(\text{0.}9\text{,0.}1\right) & \left(\text{0.}9\text{,0.}1\right) & \left(\text{0.}9\text{,0.}1\right) & \left(\text{0.}9\text{,0.}1\right) & \left(\text{0.}9\text{,0.}1\right) & \left(\text{0.}9\text{,0.}1\right) & \left(\text{0.}9\text{,0.}1\right)\\ \left(1\text{,0}\right) & \left(1\text{,0}\right) & \left(1\text{,0}\right) & \left(1\text{,0}\right) & \left(1\text{,0}\right) & \left(1\text{,0}\right) & \left(1\text{,0}\right) & \left(1\text{,0}\right) & \left(1\text{,0}\right) & \left(1\text{,0}\right) & \left(1\text{,0}\right) & \left(1\text{,0}\right) & \left(1\text{,0}\right) & \left(1\text{,0}\right) & \left(1\text{,0}\right) & \left(1\text{,0}\right) & \left(1\text{,0}\right)\\ \left(1\text{,0.}1\right) & \left(1\text{,0.}1\right) & \left(1\text{,0.}1\right) & \left(1\text{,0.}1\right) & \left(1\text{,0.}1\right) & \left(1\text{,0.}1\right) & \left(1\text{,0.}1\right) & \left(1\text{,0.}1\right) & \left(1\text{,0.}1\right) & \left(1\text{,0.}1\right) & \left(1\text{,0.}1\right) & \left(1\text{,0.}1\right) & \left(1\text{,0.}1\right) & \left(1\text{,0.}1\right) & \left(1\text{,0.}1\right) & \left(1\text{,0.}1\right) & \left(1\text{,0.}1\right)\\ \left(\text{0.}9\text{,0.}3\right) & \left(\text{0.}9\text{,0.}3\right) & \left(\text{0.}9\text{,0.}3\right) & \left(\text{0.}9\text{,0.}3\right) & \left(\text{0.}9\text{,0.}3\right) & \left(\text{0.}9\text{,0.}3\right) & \left(\text{0.}9\text{,0.}3\right) & \left(\text{0.}9\text{,0.}3\right) & \left(\text{0.}9\text{,0.}3\right) & \left(\text{0.}9\text{,0.}3\right) & \left(\text{0.}9\text{,0.}3\right) & \left(\text{0.}9\text{,0.}3\right) & \left(\text{0.}9\text{,0.}3\right) & \left(\text{0.}9\text{,0.}3\right) & \left(\text{0.}9\text{,0.}3\right) & \left(\text{0.}9\text{,0.}3\right) & \left(\text{0.}9\text{,0.}3\right)\\ \left(\text{0.}9\text{,0.}2\right) & \left(\text{0.}9\text{,0.}2\right) & \left(\text{0.}9\text{,0.}2\right) & \left(\text{0.}9\text{,0.}2\right) & \left(\text{0.}9\text{,0.}2\right) & \left(\text{0.}9\text{,0.}2\right) & \left(\text{0.}9\text{,0.}2\right) & \left(\text{0.}9\text{,0.}2\right) & \left(\text{0.}9\text{,0.}2\right) & \left(\text{0.}9\text{,0.}2\right) & \left(\text{0.}9\text{,0.}2\right) & \left(\text{0.}9\text{,0.}2\right) & \left(\text{0.}9\text{,0.}2\right) & \left(\text{0.}9\text{,0.}2\right) & \left(\text{0.}9\text{,0.}2\right) & \left(\text{0.}9\text{,0.}2\right) & \left(\text{0.}9\text{,0.}2\right)\\ \left(1\text{,0.}5\right) & \left(1\text{,0.}5\right) & \left(1\text{,0.}5\right) & \left(1\text{,0.}5\right) & \left(1\text{,0.}4\right) & \left(1\text{,0.}4\right) & \left(1\text{,0.}4\right) & \left(1\text{,0.}4\right) & \left(1\text{,0.}5\right) & \left(1\text{,0.}5\right) & \left(1\text{,0.}4\right) & \left(1\text{,0.}5\right) & \left(1\text{,0.}5\right) & \left(1\text{,0.}4\right) & \left(1\text{,0.}5\right) & \left(1\text{,0.}5\right) & \left(1\text{,0.}5\right)\\ \left(\text{0.}8\text{,0.}3\right) & \left(\text{0.}8\text{,0.}3\right) & \left(\text{0.}8\text{,0.}3\right) & \left(\text{0.}8\text{,0.}3\right) & \left(\text{0.}8\text{,0.}3\right) & \left(\text{0.}8\text{,0.}3\right) & \left(\text{0.}8\text{,0.}3\right) & \left(\text{0.}8\text{,0.}3\right) & \left(\text{0.}8\text{,0.}3\right) & \left(\text{0.}8\text{,0.}3\right) & \left(\text{0.}8\text{,0.}3\right) & \left(\text{0.}8\text{,0.}3\right) & \left(\text{0.}8\text{,0.}3\right) & \left(\text{0.}8\text{,0.}3\right) & \left(\text{0.}8\text{,0.}3\right) & \left(\text{0.}8\text{,0.}3\right) & \left(\text{0.}8\text{,0.}3\right)\\ \left(\text{0.}9\text{,0.}1\right) & \left(\text{0.}9\text{,0.}1\right) & \left(\text{0.}9\text{,0.}1\right) & \left(\text{0.}9\text{,0.}1\right) & \left(\text{0.}9\text{,0.}1\right) & \left(\text{0.}9\text{,0.}1\right) & \left(\text{0.}9\text{,0.}1\right) & \left(\text{0.}9\text{,0.}1\right) & \left(\text{0.}9\text{,0.}1\right) & \left(\text{0.}9\text{,0.}1\right) & \left(\text{0.}9\text{,0.}1\right) & \left(\text{0.}9\text{,0.}1\right) & \left(\text{0.}9\text{,0.}1\right) & \left(\text{0.}9\text{,0.}1\right) & \left(\text{0.}9\text{,0.}1\right) & \left(\text{0.}9\text{,0.}1\right) & \left(\text{0.}9\text{,0.}1\right)\\ \left(1\text{,0}\right) & \left(1\text{,0}\right) & \left(1\text{,0}\right) & \left(1\text{,0}\right) & \left(1\text{,0}\right) & \left(1\text{,0}\right) & \left(1\text{,0}\right) & \left(1\text{,0}\right) & \left(1\text{,0}\right) & \left(1\text{,0}\right) & \left(1\text{,0}\right) & \left(1\text{,0}\right) & \left(1\text{,0}\right) & \left(1\text{,0}\right) & \left(1\text{,0}\right) & \left(1\text{,0}\right) & \left(1\text{,0}\right)\\ \left(\text{0.}8\text{,0.}3\right) & \left(\text{0.}8\text{,0.}3\right) & \left(\text{0.}8\text{,0.}3\right) & \left(\text{0.}8\text{,0.}3\right) & \left(\text{0.}8\text{,0.}3\right) & \left(\text{0.}8\text{,0.}3\right) & \left(\text{0.}8\text{,0.}3\right) & \left(\text{0.}8\text{,0.}3\right) & \left(\text{0.}8\text{,0.}3\right) & \left(\text{0.}8\text{,0.}3\right) & \left(\text{0.}8\text{,0.}3\right) & \left(\text{0.}8\text{,0.}3\right) & \left(\text{0.}8\text{,0.}3\right) & \left(\text{0.}8\text{,0.}3\right) & \left(\text{0.}8\text{,0.}3\right) & \left(\text{0.}8\text{,0.}3\right) & \left(\text{0.}8\text{,0.}3\right)\\ \left(\text{0.}8\text{,0.}2\right) & \left(\text{0.}8\text{,0.}2\right) & \left(\text{0.}8\text{,0.}2\right) & \left(\text{0.}8\text{,0.}2\right) & \left(\text{0.}8\text{,0.}2\right) & \left(\text{0.}8\text{,0.}2\right) & \left(\text{0.}8\text{,0.}2\right) & \left(\text{0.}8\text{,0.}2\right) & \left(\text{0.}8\text{,0.}2\right) & \left(\text{0.}8\text{,0.}2\right) & \left(\text{0.}8\text{,0.}2\right) & \left(\text{0.}8\text{,0.}2\right) & \left(\text{0.}8\text{,0.}2\right) & \left(\text{0.}8\text{,0.}2\right) & \left(\text{0.}8\text{,0.}2\right) & \left(\text{0.}8\text{,0.}2\right) & \left(\text{0.}8\text{,0.}2\right)\\ \left(1\text{,0}\right) & \left(1\text{,0}\right) & \left(1\text{,0}\right) & \left(1\text{,0}\right) & \left(1\text{,0}\right) & \left(1\text{,0}\right) & \left(1\text{,0}\right) & \left(1\text{,0}\right) & \left(1\text{,0}\right) & \left(1\text{,0}\right) & \left(1\text{,0}\right) & \left(1\text{,0}\right) & \left(1\text{,0}\right) & \left(1\text{,0}\right) & \left(1\text{,0}\right) & \left(1\text{,0}\right) & \left(1\text{,0}\right)\\ \left(\text{0.}9\text{,0.}1\right) & \left(\text{0.}9\text{,0.}1\right) & \left(\text{0.}9\text{,0.}1\right) & \left(\text{0.}9\text{,0.}1\right) & \left(\text{0.}9\text{,0.}1\right) & \left(\text{0.}9\text{,0.}1\right) & \left(\text{0.}9\text{,0.}1\right) & \left(\text{0.}9\text{,0.}1\right) & \left(\text{0.}9\text{,0.}1\right) & \left(\text{0.}9\text{,0.}1\right) & \left(\text{0.}9\text{,0.}1\right) & \left(\text{0.}9\text{,0.}1\right) & \left(\text{0.}9\text{,0.}1\right) & \left(\text{0.}9\text{,0.}1\right) & \left(\text{0.}9\text{,0.}1\right) & \left(\text{0.}9\text{,0.}1\right) & \left(\text{0.}9\text{,0.}1\right) \end{array}\right] \end{array}$$
   where ∧ is an “and” operation that can be used in the “min” operation; ∨ is an “or” operation that can be used in the “max” operation.
Step 2: the defect level of output $\overset{´}{b}$ for the conclusion is as follows, based on Premise 2 and the formula (14), as well as the above expression (18). The fuzzy degree of membership and intuitionistic degree of nonmembership of $\overset{´}{b}=\left[\overset{´}{a}\text{ is medium}\right]{}^{\circ}\left[a\text{ is normal},\text{then }b\text{ is serious}\right]$ are as follows:
  (21) $$\begin{array}{c} \left(\mu_{M_{AT2}}\left(\overset{´}{b}\right),\nu_{M_{AT2}}\left(\overset{´}{b}\right)\right)=\left(\mu_{M_{AT1}}\left(\overset{´}{a}\right),\nu_{M_{AT1}}\left(\overset{´}{a}\right)\right){}^{\circ}F\left(a,b\right)\\ =\left(\begin{array}{c} \left(1,0\right)\left(0.3,0.4\right)\left(0.2,0.8\right)\left(0.1,0.9\right)\left(0.4,0.3\right)\left(0.3,0.4\right)\\ \left(0.3,0.7\right)\left(0.2,0.7\right)\left(0.1,0.8\right)\left(0,0.6\right)\left(0,0.9\right)\left(0.5,0.4\right)\\ \left(0.2,0.7\right)\left(0.3,0.2\right)\left(0.4,0.6\right)\left(0.2,0.5\right)\left(0.4,0.5\right){}^{\circ}F\left(a,b\right) \end{array}\right)\\ =\left(\begin{array}{c} \left(0.5,0.3\right)\left(0.5,0.3\right)\left(0.5,0.3\right)\left(0.5,0.3\right)\left(0.6,0.2\right)\left(0.8,0.1\right)\\ \left(0.6,0.3\right)\left(0.7,0.2\right)\left(0.5,0.3\right)\left(0.5,0.3\right)\left(0.6,0.3\right)\left(0.5,0.3\right)\\ \left(0.5,0.3\right)\left(0.7,0.2\right)\left(0.5,0.3\right)\left(0.5,0.3\right)\left(0.5,0.3\right) \end{array}\right). \end{array}$$

When compared to the degree (*μ*_serious_, *ν*_serious_)

(22) $$\begin{array}{c} \left(\begin{array}{c} \left(0,0.6\right)\left(0.2,0.7\right)\left(0.3,0.7\right)\left(0.4,0.5\right)\left(0.6,0.2\right)\left(0.8,0.1\right)\left(0.6,0.3\right)\left(0.7,0.2\right)\\ \left(0.1,0.7\right)\left(0.3,0.6\right)\left(0.6,0.4\right)\left(0.2,0.8\right)\left(0.1,0.9\right)\left(0.7,0.2\right)\left(0.3,0.7\right)\left(0.1,0.9\right)\left(0.2,0.8\right) \end{array}\right). \end{array}$$

of “serious” in *M*_*AT*2_, which corresponds to the fault parameters *W*_1_, *W*_2_,…, *W*_17_, the degree of $\overset{´}{b}$ in *M*_*AT*2_ is as follows:

(23) $$\begin{array}{c} \left(\begin{array}{c} \left(0.5,0.3\right)\left(0.5,0.3\right)\left(0.5,0.3\right)\left(0.5,0.3\right)\left(0.6,0.2\right)\left(0.8,0.1\right)\left(0.6,0.3\right)\left(0.7,0.2\right)\\ \left(0.5,0.3\right)\left(0.5,0.3\right)\left(0.6,0.3\right)\left(0.5,0.3\right)\left(0.5,0.3\right)\left(0.7,0.2\right)\left(0.5,0.3\right)\left(0.5,0.3\right)\left(0.5,0.3\right) \end{array}\right), \end{array}$$

which signifies “more serious.” If $\overset{´}{a}$ is a medium fault, the inference result for the output $\overset{´}{b}\in M_{AT2}$ is a more serious fault, which corresponds to objective reality.

## 6. Conclusion

Traditional HEV failure diagnostic methods are component-centric and may not explicitly incorporate communication or scheme interactions. This research assessed hardware, programming, and communication flaws in a hybrid electric vehicle's regenerative braking system (RBS) and suggested a data-driven method for discovering and identifying them. The defects investigated include parametric and sensor-related issues (underlying physical faults), software logic flaws, and interprocess communication flaws (missed messages, multiple messages, and obsolete message faults).

The intuitionistic fuzzy set (IFS) is a well-known generalization of fuzzy sets that have been thoroughly studied, with significant research into its theocratic properties and applications in various disciplines. Because nonmembership grades are involved, IFS can handle uncertainties better than fuzzy sets. In this research, the effectiveness of IFS is used to detect flaws in a regenerative braking system. First, the finite deterministic fully intuitionistic fuzzy automata (FDFIFA) are defined, and then, a semigroup over FDFIFA is designed. The algebraic properties of the FDFIFA semigroup are investigated and used to construct inference systems over it. The proposed method outperforms the previously published fuzzy inference method. Fuzzy inference can be obtained from intuitionistic fuzzy inference by considering only the membership values.

Furthermore, any machine's maximum default and present running states can be diagnosed using the maximum value of the membership and nonmembership grades. Based on the given target qualities, the current techniques must create equations or expressions to deal with the target. The described approach, on the other hand, uses its state transition mapping to execute characteristic processing and just requires the selection of system parameters. There are a number of practical generalizations of fuzzy sets [9, 61–68], and inference rules for these generalizations can be developed using the same techniques. The proposed methodology's superiority is demonstrated by the real-life example, which accurately and efficiently discovers the defect. The proposed methodology can be used to detect a failure in any machine by identifying its critical components, the factors that can cause any fault in those components, and the fault caused by these parameters. The nature and severity of the defect can be used to award membership and nonmembership grades.

## Figures and Tables

**Figure 1:** Fully intuitionistic fuzzy state transition.

**Figure 2:** Fully intuitionistic fuzzy state transition.

**Figure 3:** Series-parallel power train.

**Table 1:** Mapping effects on states.

*∗*	*f*_∧_	*f*_*e*_1__	*f*_*e*_2__
*t*_1_	*t*_1_	*t*_1_	*t*_3_
*t*_2_	*t*_2_	*t*_1_	*t*_3_
*t*_3_	*t*_3_	*t*_2_	*t*_3_

**Table 2:** Composition of mappings.

°	*f*_∧_	*f*_*e*_1__	*f*_*e*_2__
*f*_∧_	*f*_∧_	*f*_*e*_1__	*f*_*e*_2__
*f*_*e*_1__	*f*_*e*_1__	*f*_*e*_1_ *e*_1__	*f*_*e*_2_ *e*_1__
*f*_*e*_2__	*f*_*e*_2__	*f*_*e*_2__	*f*_*e*_2__

## Data Availability

Data are collected from relevant stakeholders through questionnaire.
